# Analysis of Prevalence, Influencing Factors, and Countermeasures of Short Stature in Children and Adolescents Aged 6∼14 in Furong District, Changsha City, in 2020

**DOI:** 10.1155/2021/3933854

**Published:** 2021-08-06

**Authors:** Yanyan Li, Yun Chen, Xuan Xu, Boyu Tan, Yingbo Liu, Xuan Peng, Danxia Peng, Shuping Liu, Jinghui Yao

**Affiliations:** ^1^Department of Pediatric Endocrinology, Genetic Metabolism and Cardiology, Hunan Provincial People's Hospital (The First Affiliated Hospital of Hunan Normal University), No. 61, Liberation West Jiefang Road, Furong District, Changsha 410006, Hunan, China; ^2^Department of Pediatric Orthopedics, Center for Orthopaedic Surgery, The Third Affiliated Hospital of Southern Medical University, Guangzhou 510630, Guangdong, China

## Abstract

In recent years, children's and adolescents' growth and development issues have received increasing attention with the socioeconomic development. The etiology of child short stature involves heredity, race, sex, nutrition, and a variety of endocrine hormones, which is very complex. The age of 6∼14 is the key period of children's development. Understanding the height characteristics, the prevalence of short stature, and its influencing factors at this stage and formulating preventive measures as soon as possible are conducive to improving the average height of children and reducing the incidence of short stature. In this study, cluster sampling was used to select 56,865 children and adolescents aged 6∼14 years old from 40 primary and secondary schools in Furong District of Changsha City, and the height of each child and adolescent was measured. The results showed that the overall crude prevalence of short stature in children aged 6∼14 in Furong District of Changsha is 2.82%. Growth hormone level <10 *μ*g/L, pubertal retardation, familial short stature, low egg intake, and intrauterine growth retardation are independent risk factors affecting the occurrence of short stature. In order to improve the status quo of short stature of children aged 6∼14 in Furong District, Changsha City, targeted intervention should be strengthened for people with combined high risk factors.

## 1. Introduction

Short stature (SS) refers to children of the same race, sex, and age whose height is 2 standard deviations lower than the average height of normal population or lower than the 3rd percentile in similar living environment, which is a common disease in pediatrics [1]. Epidemiology shows that the total detection rate of short stature in children in Suzhou area is 2.89%, the prevalence rate of short stature in children in Wuhan is 5.47%, and that in Yizheng was 2.2% [2]. It can be seen that the incidence of short stature in children in China is high. Studies have found that short stature will not only affect the height of children but also lead to varying degrees of behavioral adaptation disorder, stunted puberty, mental retardation, and psychological barrier [3]. In addition, the incidence of chronic cardiopulmonary insufficiency and neurological dysfunction in children will also increase. Therefore, it is of great significance to diagnose short stature as early as possible and give appropriate and systematic treatment according to the etiology to improve the clinical symptoms and improve the quality of life of children.

The etiology of short stature in children is complex and involves genetics, race, gender, nutrition, and various endocrine hormones [4]. In order to further clarify the prevalence of short stature among children and adolescents in Furong District of Changsha, this study investigated the height distribution characteristics of primary and middle school students in this area and analyzed possible risk factors in order to provide scientific basis and countermeasures for clinical treatment.

## 2. Materials and Methods

### 2.1. General Information

A total of 56,865 students aged 6∼14 from 40 primary and secondary schools in Furong District of Changsha were selected as the research objects from September to October, 2020, by cluster sampling method. Each person issued a questionnaire on factors related to short stature, a total of 56,865 copies were issued.

### 2.2. Inclusion Criteria

(i) The age of 6∼14 years old; (ii) with no congenital organ loss; (iii) sound limbs; (iv) Han nationality; (v) the permanent resident population of Furong District, Changsha City.

### 2.3. Exclusion Criteria

(i) Diseases affecting growth and development, such as digestive system diseases, urinary system diseases, and iron deficiency anemia; (ii) mental retardation; (iii) patients who were administrated with drugs that inhibited bone marrow or erythropoietin within six months before enrollment; (iv) patients who had heart, brain, liver, kidney, and other vital organ dysfunction.

### 2.4. Method

#### 2.4.1. Collecting the Data

Parents completed the questionnaires based on the content of the survey and the specific circumstances of their own children. The main investigation contents included paternal height, maternal height, the manner of delivery, birth weight, the history of genetic diseases, egg intake, milk intake, meat intake, sleep time at night, and weekly exercise frequency.

#### 2.4.2. Physical Examination Requirements

The physical examination was conducted according to the Project of Health Checklist for Primary and Middle School Students [5]. The method of height measurement referred to the requirements of National Standards for Students' Physique [6]and Administrative Measures for Physical Examination of Primary and Secondary School Students [7]. The testee must take off his/her shoes when measuring the height. The requirements for the posture include standing upright, keeping head, hip, and heel abut against the measuring column at three points, and looking ahead with both eyes. The height of all study subjects is the average of 3 repeated measurements, and the reading must be accurate to 0.1 cm.

### 2.5. Diagnostic Criteria for Short Stature [8]

If the following two or more indicators are met, it can be diagnosed as short stature: (i) the height being lower than the average height of normal people by 2 standard deviations. (ii) The imaging test showing that the bone age is more than 2 years behind the actual bone age. (iii) The level of growth hormone being less than 10 *μ*g/L. (iv) Height increased by less than 5.0 cm/year. (v) Turner syndrome. (vi) Hypothyroidism. (vii) The average height of parents being less than 155.0 cm.

### 2.6. Statistical Methods

All data were processed with SPSS 22.0 statistical software, and GraghPad prism 8 was used to make statistical graphs. In order to ensure the accuracy of the data, double entry was recorded during the survey. Measurement data are expressed as mean ± standard deviation ($\bar{x}$ ± s), independent sample *t*-test is used for comparison between groups, count data is expressed as (*n* (%)), and chi-square (*χ*^2^) test is performed. Multivariate logistic regression model was used to analyze the related factors affecting the short stature in children. The difference is statistically significant when *P* < 0.05.

## 3. Results

### 3.1. Basic Situation

In this study, a total of 56,865 primary and secondary school students were sampled and investigated, of which 2,848 were younger than 6 or older than 14 years old, 243 were incomplete for height information filling, and 53,772 were finally included after exclusion.

### 3.2. Height Distribution Characteristics of Various Age Groups

The average height of male students in the age group of 6∼8 is higher than that of female students. The average height of female students in the age group of 9∼11 is slightly higher than that of male students. The average height of male students in the age group of 12∼14 surpasses that of female students, as shown in Figure 1.

### 3.3. Comparison with National Student Physical Health Survey Results in 2014

The results of this survey show that the average height of middle school students aged 6∼14 in Furong District has little difference with the average height of the national students in 2014. The average height of 12∼14 years old group in Furong District is slightly higher than the national average height of students, and it was more obvious in the group of boys (Table 1).

### 3.4. Crude Prevalence of Short Stature

A total of 1,517 of 53,772 primary and middle school students suffer from short stature, and the overall crude prevalence rate of short stature is 2.82%. Among them, the prevalence rate of male short stature was 2.62%, while that of female was 3.05%, and there was no statistical difference between male and female groups (*P* > 0.05) (Table 2).

### 3.5. Univariate Analysis of Occurrence of Short Stature

Univariate analysis showed that the age, intrauterine growth retardation, maternal height, and daily milk intake in the diseased group were not statistically significant compared with those of the nondiseased group (*P* > 0.05). But there were differences in gender, growth hormone level, pubertal retardation, hypothyroidism, the occurrence of Turner syndrome, familial short stature, paternal height, egg intake, exercise status, and the occurrence of intrauterine retardation between the disaffected group and the nondiseased group (*P* > 0.05) (Table 3).

### 3.6. Variable Assignment

Whether short stature occurred was taken as the dependent variable, and the factors with significant differences in Table 3 were taken as the independent variables to be included in the logistic regression model. The assignment of the dependent variables and independent variables is shown in Table 4.

### 3.7. Multivariate Analysis of Occurrence of Short Stature

Growth hormone level <10 *μ*g/L, pubertal retardation, familial dwarfism, low egg intake, and intrauterine growth retardation were independent risk factors for dwarfism (*P* > 0.05) (Table 5).

## 4. Discussion

Height is derived from the longitudinal growth index of human body, which is influenced by heredity, nutrition, sleep, sports, living environment, living habits, race, etc. [9]. In this study, the average height of girls at the age of 9∼11 was higher than that of boys at the age of 9∼11 in Furong District of Changsha City, and the average height of boys at the age of 12∼14 surpassed that of girls. This phenomenon accords with general physiology, growth, and development rule. Due to the inability to obtain the standard deviation of each age group in the country and the inability to calculate the statistical parameter values, the difference values were compared with the results of the National Student Physical Health Survey in 2014. The results show that the average height of male schoolchildren in the age group of 12∼14 years was slightly higher than the national average height of schoolchildren in the corresponding age range, and the female group had a slightly higher average height than the national level at the age of 10∼14 years.

Short stature is a common public health problem in developing countries. Our study conducted a statistical analysis on the prevalence of dwarfism among primary and middle school students aged 6∼14 in Furong District, Changsha City. The results showed that the gross prevalence rate of short stature was 2.82%, which was significantly lower than that of short stature published by WHO in developing countries (32.5%) [10]. It is also lower than the overall prevalence of short stature in Shanghai (3.77%) [11], Wuhan (5.47%) [12], and Rong'an County (8.0%) [13], which may be closely related to genetics, regional economic level, ethnicity, dietary nutrition, endocrine hormone levels, and other factors.

Short stature not only causes physical deficits in the affected children but also brings great psychological impact on children, which is not conducive to healthy growth [14]. The result of our study showed that growth hormone level <10 *μ*g/L, pubertal retardation, familial dwarfism, low egg intake, and intrauterine growth retardation were independent risk factors for dwarfism (*P* > 0.05). Reasons for this include the following: (i) the growth hormone receptor gene is closely related to the occurrence of short stature. Previous studies have shown that the growth hormone receptor gene mutation will affect the growth hormone and the receptor binding, and then cause signaling disorders, affect the function of growth hormone, and impede growth and development [15]. (ii) Adolescent developmental delay, which means that no secondary sexual characteristics appear at the age of 13 in girls or 14 in boys, may affect height development to some extent [16]. (iii) Inheritance is decisive for child growth and development, and individuals with short stature in an immediate family have a much higher incidence of this condition than those without a family history of short stature [17]. (iv). The acquired nutrition intake is the key to determine the growth and development of children. Eggs are rich in high-quality protein groups, which contain amino acids such as leucine, isoleucine, lysine, and methionine, which can maintain life and growth [18]. (v). Full-term infants with body weight less than 2,500 g or birth length less than 47 cm are defined as having intrauterine growth retardation. Studies suggest that the population which has growth-related endocrine abnormalities and insensitivity to growth hormone has a much higher chance of developing short stature in childhood than in normal population [19].

There are many drugs for short stature, including recombinant human growth hormone (rhGH), gonadotropin-releasing hormone analogs (GnRHA), aromatase inhibitors (AI), insulin-like growth factor 1 (IGF-1), protein assimilation hormones, and traditional Chinese medicine [20]. However, there is no uniform protocol for the treatment of short stature at present, so it is necessary to develop a series of preemptive measures. First of all, the relevant institutions need to strengthen the education of knowledge related to prenatal and postnatal care. They must actively carry out prenatal screening, promote prenatal genetic diagnosis, and avoid the birth of children with genetic tendency of short stature as far as possible. Secondly, pregnant women need to strengthen nutrition during pregnancy to avoid the birth of children with intrauterine growth retardation due to malnutrition. Most importantly, it is necessary to carry out health education for people with combined risk factors and advocate them to keep scientific diet habits, and actively exercise, and then promote growth and development.

Due to the limitation of research conditions, this study only conducted a general survey of primary and middle school students in Furong District, and the results of cluster sampling may be slightly higher than random sampling. Therefore, the results of this study may not be fully representative of the overall situation of primary and secondary school students in the whole urban area of Changsha, so the results should be interpreted with caution. In summary, the overall crude prevalence of short stature in children aged 6∼14 in Furong District of Changsha is 2.82%. Growth hormone level <10 *μ*g/L, pubertal retardation, familial short stature, low egg intake, and intrauterine growth retardation are independent risk factors affecting the occurrence of short stature. In order to improve the status quo of short stature of children aged 6–14 in Furong District, Changsha City, targeted intervention should be strengthened for people with combined high risk factors.

## Figures and Tables

**Figure 1:** Height distribution characteristics of various age groups. The average height of male students in the age group of 6∼9 is higher than that of female students. The average height of female students in the age group of 9∼11 is slightly higher than that of male students. The average height of male students in the age group of 12∼14 surpasses that of female students.

**Table 1:** Comparison of average height of 6–14-year-old primary and middle school students in Furong District of Changsha City in 2020 and national student physical health data in 2014 (cm).

Group	Average height of males			Average height of females		
	Furong District	National	*D*-value	Furong District	National	*D*-value
6∼6.9	120.66	119.7	0.96	119.10	118.1	1.00
7∼7.9	126.09	126.6	−0.51	124.77	125.1	−0.33
8∼8.9	131.55	132.0	−0.45	130.60	130.5	0.10
9∼9.9	137.10	137.2	−0.10	137.05	136.3	0.75
10∼10.9	142.44	142.1	0.34	143.98	142.6	1.38
11∼11.9	148.78	148.1	0.68	150.24	149.3	0.94
12∼12.9	155.86	154.5	1.36	155.10	153.7	1.40

**Table 2:** Crude prevalence rate of short stature in boys and girls of different age groups in Furong District, Changsha, in 2020 (*n*, %).

Group	Males	Females	Prevalence rate	*χ* ^2^	*P* value
6	69/3545 (1.95%)	127/3213 (3.95%)	196/6758 (2.9%)	24.09	1.00
7	92/4020 (2.29%)	133/3694 (3.6%)	225/7714 (2.92%)	11.70	0.999
8	97/4275 (2.27%)	122/3692 (3.3%)	219/7967 (2.75%)	7.95	0.995
9	92/3708 (2.48%)	99/3312 (2.99%)	191/7020 (2.72%)	1.71	0.808
10	119/3658 (3.25%)	89/3246 (2.74%)	208/6904 (3.01%)	1.54	0.785
11	115/3650 (3.15%)	59/2917 (2.02%)	174/6567 (2.65%)	8.00	0.995
12	80/2080 (3.85%)	31/1771 (1.75%)	111/3851 (2.88%)	15.01	1.00
13	86/3721 (2.31%)	107/3270 (3.27%)	193/6991 (2.76%)	5.98	0.985

**Table 3:** Univariate analysis of occurrence of short stature.

Clinical information	Diseased group (*n* = 1517)	Nondiseased group (*n* = 52255)	*χ* ^*2*^ */t*	*P* value
Gender				
Male	750 (49.44)	27817 (53.23)	8.938	0.003
Female	767 (50.56)	24348 (46.59)		
Age (years old)	9.41 ± 2.31	9.36 ± 2.39	0.804	0.421
Growth hormone level				
＜10 *μ*g/L	1026 (67.63)	12109 (23.17)	1578.586	0.000
≥10 *μ*g/L	491 (32.37)	40146 (76.83)		
Pubertal retardation				
Yes	1043 (68.75)	10374 (19.85)	21007.933	0.000
No	474 (31.25)	41881 (80.15)		
Intrauterine growth retardation				
Yes	59 (3.89)	2103 (4.02)	0.070	0.792
No	1458 (96.11)	50152 (95.98)		
Hypothyroidism				
Yes	549 (36.19)	65989 (12.63)	710.231	0.000
No	968 (63.81)	45657 (87.37)		
Turner syndrome				
Yes	161 (10.61)	1173 (2.24)	426.718	0.000
No	1356 (89.39)	51082 (97.76)		
Familial short stature				
Yes	992 (65.39)	6149 (11.77)	3681.029	0.000
No	525 (34.61)	46106 (88.23)		
Paternal height	156.56 ± 14.37	173.41 ± 16.79	38.679	0.000
Maternal height	150.36 ± 10.12	150.42 ± 10.69	0.216	0.829
Egg intake				
Occasionally or not	571 (37.64)	3054 (5.84)	2791.266	0.000
Less than once a week	454 (29.93)	8616 (16.49)		
1–2 times a week	296 (19.51)	17119 (32.76)		
3–5 times a week	196 (12.92)	23466 (44.91)		
Daily milk intake				
＜250 mL	491 (32.37)	17471 (33.43)	4.590	0.101
250–500 mL	546 (35.99)	17440 (33.37)		
＞500 mL	480 (31.64)	17344 (33.19)		
Exercise status				
Never	175 (11.54)	5413 (10.36)	39.989	0.000
≤1 times	378 (24.92)	9946 (19.03)		
2–3 times	426 (28.08)	15679 (30.00)		
≥4 times	538 (35.46)	21217 (40.60)		

**Table 4:** Variable assignment table.

Variable	The assignment
Dependent variable	
Short stature	No = 0, yes = 1
Independent variables	
Gender	No = 0, yes = 1
Growth hormone level	<10 *μ*g/L = 0, ≥10 *μ*g/L = 1
Pubertal retardation	No = 0, yes = 1
Hypothyroidism	No = 0, yes = 1
Turner syndrome	No = 0, yes = 1
Familial short stature	No = 0, yes = 1
Egg intake occasionally or not	1∼2 times a week or 3∼5 times a week = 0, occasionally or not or less than once a week = 1
Exercise status never or once in a while	2∼3 times or ≥4 times = 0, never or ≤1 times = 1
Paternal height	Input as actual height
Intrauterine growth retardation	No = 0, yes = 1

**Table 5:** Multivariate analysis of occurrence of short stature.

Factors	*β*	SE	Wald *χ*^*2*^	*P* value	OR	OR 95% CI
Gender	2.354	2.643	25.656	0.591	16.2621	0.349–6.318
Growth hormone level <10 *μ*g/L	3.519	0.474	26.216	0.000	20.593	4.599–1.379
Pubertal retardation	1.374	0.243	12.262	0.000	6.891	1.896–1.064
Hypothyroidism	1.256	1.135	11.953	0.064	6.159	0.948–4.565
Turner syndrome	1.065	1.158	11.049	0.071	6.005	0.285–8.351
Familial short stature	0.346	0.291	0.479	0.000	0.874	1.463–1.258
Egg intake occasionally or not	0.686	0.176	0.716	0.000	0.943	1.634–1.279
Exercise status never or ≤1 times	0.169	0.436	0.297	0.504	0.346	0.341–1.588
Paternal height	−0.907	0.359	20.695	0.132	0.163	0.476–2.154
Intrauterine growth retardation	1.676	0.474	10.595	0.000	7.198	1.956–1.533

## Data Availability

The datasets used and analyzed during the current study are available from the corresponding author and the first authors on reasonable request.
